The article "Web Log Analysis and Security Assessment Method Based on Data Mining" was published in 2022. Journal: Comput Intell Neurosci.

# Web Log Analysis and Security Assessment Method Based on Data Mining

**DOI:** 10.1155/2022/8485014

**Published:** 2022-08-25

**Authors:** Jingquan Jin, Xin Lin

**Affiliations:** ^1^Computer Department, Anhui Post and Telecommunication College, Hefei 230031, China; ^2^Department of Information Technology, Anhui Vocational College of City Management, Hefei 230011, China

## Abstract

Web content mining describes the classification, clustering, and attribute analysis of a large number of text documents and multimedia files on the web. Special tasks include retrieval of data from the Internet search engine tool W; structured processing and analysis of web data. Today's blog analysis has security concerns. We do experiments to investigate its safety. Through experiments, we draw the following conclusions: (1) Web log extraction can use efficient data mining algorithms to systematically extract logs from web servers, then determine the main access types or interests of users, and then to a certain extent, based on the discovered user patterns, analyze the user's access settings and behavior. (2) No matter in the test set or the mixed test set, the curve value of deep mining is very stable, the curve value has been kept at 0.95, and the curve value of fuzzy statistics method and quantitative statistics method is stable within the interval of 0.90–095. The results also show that the data mining method has the highest identification accuracy and the best security performance. (3) Web usage analysis requires data abstraction for pattern discovery. This data abstraction can be achieved through data preprocessing, which introduces different formats of web server log files and how web server log data is preprocessed for web usage analysis. One of the most critical parts of the web mining field is web log mining. Web log mining can use powerful data mining algorithms to systematically mine the logs in the web server and then learn the user's access or preferred interests and then conduct a certain degree of user preferences and behavior patterns according to the discovered user patterns. Based on the above analysis, the current web log analysis is faced with security problems. We conduct experiments to study to verify the security performance of web logs and draw conclusions through experiments.

## 1. Introduction

Methods developed since the 1970s to represent, process, and extract knowledge for a variety of applications from the ever-increasing accumulation of data have made the pervasiveness of computing possible, perhaps inevitable, and have built a system for examining and a general framework for classification methods. Provide simple examples to demonstrate the nature of representative feature selection methods, compare them using datasets with a combination of intrinsic properties according to the goal of selecting features, propose guidelines for using different methods in various situations, and identify areas of research new challenge venue. There is a reference for researchers in machine learning, data mining, knowledge discovery, or databases [1]. As the ability to track and collect large amounts of data using current hardware technologies continues to improve, there is a lot of interest in developing data mining algorithms that protect users. Recently proposed approaches have addressed data protection issues by aggregating data and restoring aggregation level distributions for data mining. This technology protects the confidentiality of the information contained in the original mark. Of course, rebuilding a distribution will result in an acceptable loss of information in many real situations. The algorithm is better in terms of data loss levels than currently available methods. In particular, the EM algorithm has been shown to satisfy the maximum likelihood method of the initial distribution in noise-based estimation. When large amounts of data are available, the EM algorithm provides a reliable estimate of the raw data [2]. Interest in mining time series data has exploded over the past decade. In this work, the following claims are made. Much of the utility of this work is small, because the amount of improvement provided by the contributions is entirely the variance that can be observed by testing on many real-world datasets or by changing minor implementation details. To illustrate this point, the most exhaustive time series experiment ever performed has been reimplemented [3]. The Bayesian network is a graphical model that encodes probability relationships between variables of interest. When used in statistical methods, the model has many advantages in data modeling because it encodes relationships between all variables, facilitates the processing of missing data, and can be used to understand problems and predict results. This article describes the construction of the Bayesian network based on historical data and summarizes Bayesian statistical methods for using the data to improve these models [4]. The use of soft-computing provides an overview of the available data mining literature. Classifications were made based on the various software computing tools used and the data mining activities they performed, as well as the data mining activities performed and the preference criteria selected of the model. The utility of various soft computation methods is emphasized. In general, fuzzy sets are useful for solving problems related to image comprehension, mixed-media information, and human interaction and can provide approximate solutions more quickly. Genetic algorithms provide efficient search algorithms for selecting models from mixed-media data, pointing out specific problems for data mining, and applications of soft-computing techniques are presented in extensive bibliography [5]. Access blogs through business services and academic research are usually limited to the content of web posts. In this paper we provide a large-scale study of blogging and its relationship to posts. Using a large-scale comment corpus, we estimate the large number of comments in the blogosphere; analyze the relationship between blog popularity and comment patterns; and measure the contribution of comment content to various aspects of our blog visits [6]. Several systems have been developed to provide statistical analysis of World Wide Web usage logs. These programs typically report the number of files used and the number of times the site was used by the site, and some programs even provide time-of-request analysis. However, these programs are not interactive and cannot see the local database. The Internet is designed to provide database administrators and designers with graphical representations and templates for accessing local databases. In other words, by incorporating the network path paradigm into interactive software, users can not only view documents in the database, but also contact users by requesting documents from the database [7]. It presents the methods and analysis used in the ongoing, three-year Excite research project, which aims to examine the search nature of major Internet search engines. This article starts with general information about the web, unique and attractive views of users searching the web, and the impact of the web. The main content of this article discusses the structures and methods used so far in material analysis and concludes with conclusions and expectations for future network research [8]. Web usage analysis or web usage analysis or web log extraction or clickthrough rate analysis is the process of extracting useful information from web server logs, database logs, user requests, client-side cookies, and user profiles to test the performance of web users. Internet usage analysis requires data abstraction to find patterns. This data abstraction can be achieved by data preprocessing, which adopts different web server log file formats and how the web server log data is preprocessed to analyze network usage [9]. Log files are maintained in communication between web browsers and web servers generated by real users accessing content associated with dynamic hyperlinks. These log files represent past user access to content and are used to generate web crawler access. This approach allows crawlers to accurately simulate real users, leading to the ability of legacy bots to automatically access everything a real user can access [10]. A method of evaluating an organization's information security policies and practices, including identifying risks associated with information security policies and practices, collecting information about information security policies and practices, using a security due date assessment matrix, generating ratings from the collected information, and correlating information with information risks associated with security policies and exercises, is to use ratings to generate a list of corrective actions, execute the list of corrective actions to create new security information policies and exercises, and monitor new security information policies and exercises [11]. Ecological security is a challenging issue for human survival and development. Cities are efficient and interactive human activities, resource shortages prevent further urban development, and ecological refugees and environmental health issues affect human survival. Urban ecological security is threatening the sustainable development of cities. There is an urgent need to appreciate urban sustainability. There is an urgent need to appreciate that urban ecological security and urban ecological security assessment are the most important issues. Through the assessment, decision makers can obtain more information about the current status of urban ecological security so that they can issue rational strategies to solve the problem. People can obtain information in time and then take decisive action to protect themselves [12]. Security analysis is a complex system development. The latest security scanning tools are only used to scan and detect vulnerabilities in network systems. Systems engineering thinking and techniques are applied to a comprehensive cybersecurity analysis. An artificial neural network model for safety analysis has been proposed, and computer simulation experiments have been carried out. The results show that the model can be effectively used to comprehensively evaluate the network security level. The overall assessment of the security status of computer networks provides new ideas and methods [13]. Security assessment is a complex system engineering. Through the hierarchical analysis process, various factors affecting network security are deeply studied, and a comprehensive network security ranking index system is established. A security assessment is proposed, which provides a new idea and method for the overall assessment of computer network security status [14]. Network security analysis is a complex system design. The latest security analysis tools are only used to scan and detect security vulnerabilities in network systems. Comprehensive analysis of system design and techniques applied to cybersecurity is done. Build a comprehensive evaluation index system for network security. An artificial neural network model for safety assessment is proposed, and computer simulation experiments are carried out. The results show that the model can be effectively used to comprehensively evaluate the network security level. The overall assessment of the security status of computer networks provides new ideas and methods [15].

The article "Web Log Analysis and Security Assessment Method Based on Data Mining" was published in 2022. Journal: Comput Intell Neurosci.

## 2. Web Log Analysis under Data Mining

### 2.1. Overview of Web Log Mining

Web mining is one of the most important components of the web mining industry. The web systematically extracts logs from web servers using powerful data mining algorithms to obtain information about user availability or priority of interest and is based in part on detected user patterns. Evaluate your website, adjust its topology, improve system performance, improve your website experience, provide intelligent personalization, and increase user loyalty. Internet communication is usually done through a web server architecture. The server for each site generates logs, the web client generates log files for clients accessing multiple sites, the proxy server generates log files for multiple users accessing multiple sites through a proxy, and the web server generates journal log files. Log files for multiple users using the site. Therefore, recording user habits can also capture user habits from three perspectives: network client, proxy server, and web server. Since the log information of the three nodes is different, the available user information is also different. Currently, two main aspects of the weblog algorithm are being analyzed, pattern sequence analysis algorithms and clustering algorithms. Customer usage patterns and agency buying should start online. Periodic pattern analysis algorithms are usually chosen to analyze the user's desired path, capture the content of interest to the user, and use an intelligent search engine to improve performance. Server-side clustering algorithms are commonly used to aggregate log data generated by all users visiting a website and create blogs that evaluate user behavior based on the clustering results. Finally, in this article, we will look at campus website logs to determine patterns of visitors. Therefore, it was decided to use a clustering algorithm to extract server-side access patterns.

### 2.2. Web Log Mining Process

In general, the journal launch process is divided into four steps: collecting journals, defining journals, defining templates, and modifying templates. (1) This article also uses this type of logs to review work, and there are ways to collect logs using JavaScript scripts on our web page. (2) Log preprocessing phase after the general data exploration phase; initial data preprocessing will be performed in this phase. The log data source is irregular, impure, invalid data. Raw logs are used to cover data processing. It is converted into a format suitable for intelligence assessment, stored in a single format, and then continuously assessed. (3) Use a variety of data mining algorithms according to other business needs, mainly covering cluster analysis, association recommendation, path and intelligent sequence data analysis, etc. (4) Model analysis step: This step is the process of defining and analyzing data mining, which makes the generated model easy to understand. In the case of solving fundamental problems, theoretical theory is based on the definition of strategies. The web log mining process is shown in Figure 1.

The article "Web Log Analysis and Security Assessment Method Based on Data Mining" was published in 2022. Journal: Comput Intell Neurosci.

### 2.3. Web Data Mining Classification and Development Design Focus

Web content mining involves classifying, grouping, and analyzing connections between multiple text and multimedia files on the Internet. Specific tasks include retrieving information from W search engines on the Internet; structuring and analyzing network data; page content analysis based on HTML technical standards and efficient data analysis. The implementation methods of web content extraction are mainly divided into direct document content decompression object; search engine query data retrieval object. According to different data mining objects, online content decompression includes two categories: online document decompression and media decompression. Web analysis is basically the process of searching and refining information about the structure and informational associations of pages on the World Wide Web. Its traditional implementation is as follows: First, the topology structure of the World Wide Web is analyzed using graph theory and transformed into a directed graph model. Each web page acts as a structural cue for a directed graph, with each edge of the graph representing links between different web pages. Examining the network structure can capture the necessary elements of directed graphs transformed from the World Wide Web to objects and extract valuable information from them. The purpose of a preliminary analysis of the site structure is to support search engines and provide users with valid information on the man pages. The object of web data mining research is shown in Figure 2.

The article "Web Log Analysis and Security Assessment Method Based on Data Mining" was published in 2022. Journal: Comput Intell Neurosci.

Web content mining refers to the classification, clustering, and association analysis of a large number of text documents and multimedia files on the web. The specific tasks include extracting data information from the W search engine tool in the Internet; performing structured processing and analysis on network information; analyzing the page content based on HTML technical standards and mining the effective data information.

Pure log mining analysis extracts the access records stored by the server when users access network resources. The information stored in the web log includes the user's access method, access date and time, user query, user's smart address, etc. Statistical analysis of this information allows us to examine the relationship between this information so that we can still find some key characteristics of user behavior. The key points of the development and design of network log extraction technology are as follows: (1) Before data mining, the target data must be preprocessed to meet the requirements of data mining and retrieval and to improve the level of efficient use of data. (2) OLAP can be used to perform multilevel analysis on the web log database to determine the N most popular web pages that will be opened when N users open web pages, so that users can understand their usage preferences and lay a foundation for this, so as to tap potential demand and market development.

## 3. Web Log Analysis under Data Mining Algorithm

### 3.1. Data-Based Mining Model

When performing data analysis based on historical data, data analysis can be carried out from a mathematical point of view and in accordance with the idea of time series analysis. When analyzing historical data, the algorithm used in this paper is support vector machine. Define a training set (*X*_*i*_, *Y*_*i*_) of number *n* and a nonlinear map *ψ*(*X*) as

(1) $$\begin{array}{c} \left\{\left(X_{i},Y_{i}\right)i=1,2,\ldots n\right\},\\ \psi \left(X\right)=\left(\varphi \left(x_{1}\right),\varphi \left(x_{2}\right),\ldots \varphi \left(x_{n}\right)\right). \end{array}$$

The two complete the mapping from the sample input space to high-dimensional features by a linear regression function:

(2) $$\begin{array}{c} f\left(x_{t}\right)=\omega^{T}\varphi \left(x_{t}\right)+b. \end{array}$$

Among them, *w* is the weight vector in the high-dimensional space, and *b* is the bias of the model. The ultimate goal of the SVM algorithm is to minimize the structural risk, that is, to find the optimal *w* and *b*. During the calculation of model parameters, SVM is usually based on the principle of structural risk minimization:

(3) $$\begin{array}{c} \min J=\frac{1}{2}\omega^{2}+c\sum_{i=1}^{n}\left(\xi_{i}+\xi_{l}\right)\\ s.t\left\{y_{i}-\omega^{T}\varphi \left(x_{i}\right)-b\leq \varepsilon +\xi_{i}.\right) \end{array}$$

Among them, *c* is the regularization coefficient in the optimization process, and *ξ*_*i*_ ` *ξ*_*l*_ is the relaxation factor to adjust the structural risk. When solving the optimization problem, this paper uses the Lagrange function, and its basic process is as follows:

(4) $$\begin{array}{c} L=\frac{1}{2}\omega^{2}++c.\sum_{i=1}^{n}\left(\xi_{i}+\xi_{l}\right)-\sum_{i=1}^{n}\partial_{l}. \end{array}$$

According to the optimization algorithm there are

(5) $$\begin{array}{c} \frac{\partial L}{\partial \omega }=0⟶\omega =\sum_{i=1}^{n}\left(\alpha_{l}-\alpha_{l}\right)\varphi \left(x_{l}\right). \end{array}$$

At this point, the kernel function that defines the heap function used in the optimization process is

(6) $$\begin{array}{c} k\left(x_{i},x_{j}\right)=\varphi {\left(x_{i}\right)}^{T}\varphi \left(x_{J}\right). \end{array}$$

Finally, the prediction formula of the model can be obtained:

(7) $$\begin{array}{c} f\left(x\right)=\sum_{i=1}^{n}\left(\alpha_{l}-\alpha_{l}\right)K\left(x_{i},x_{j}\right)+b. \end{array}$$

Among them, *k*(*x*_*i*_, *x*_*j*_) is the radial basis function used in the model prediction, and its form is as follows:

(8) $$\begin{array}{c} k\left(x_{i},x_{j}\right)=\exp\left[\frac{-x_{i}-x_{j}}{2\sigma^{2}}\right]. \end{array}$$

The article "Web Log Analysis and Security Assessment Method Based on Data Mining" was published in 2022. Journal: Comput Intell Neurosci.

### 3.2. Realize Intelligent Data Mining

Use neural network technology, an important branch of artificial intelligence technology, to achieve the goal of big data mining in the Internet of Things. A BP neural network with a three-layer transmission structure is used as the main structure, and normalized data is inputted into the neural network. Due to the peculiarities of the structure of the neural network, to replace the weight of the connection between the input and intermediate layers of the network *W*, the average information-information entropy *E* is used. The formula for calculating the weight:

(9) $$\begin{array}{c} \omega =\frac{1-H_{i}}{\sum_{i=1}^{E}H_{i}}. \end{array}$$

In the formula, the calculation result of the connection weight of the neural network is obtained through the entropy value of the i-th dimension attribute of the data. A genetic learning step is added to design a classifier with the network nonlinear classification ability and network structure as the core. Through the optimization of the genetic learning algorithm, the data that meets the mining requirements is output. The improvement of this artificial intelligence technology method, while ensuring the nonlinear ability, is connected with the previous processing method to ensure the accuracy of data mining. The genetic algorithm is integrated in the data mining process, and it is necessary to complete the modification of the hybridization operator and the mutation operator on the data input to the neural network. The calculation of the hybridization operator is expressed as a linear combination, expressed as:

(10) $$\begin{array}{c} \theta_{1}=u\theta_{1}+\left(1-u\right)\theta_{2},\\ \theta_{2}=u\theta_{2}+\left(1-u\right)\theta_{1}. \end{array}$$

In the formula, *θ*_1_ and *θ*_2_ are the two data pieces of linear combination, and the value range of the constant *U* is between 0 and 1, and the value range is narrowed according to the actual situation. When the constant value is in a fixed state, it means that the hybridization operator in the calculation process is inconsistent. When the constant value changes with the number of iterations, the average performance of the hybridization operator can be improved, so that the IoT big data can be gradually mixed. In the modification of mutation operator in data mining, each random data *C* may have a certain probability of mutation, and the value Vk after one mutation of the data is randomly expressed as

(11) $$\begin{array}{c} v_{k}=v_{k}=\Delta \left(t,v_{k}-LB\right). \end{array}$$

Generate data variation values based on the left and right neighbors LB and UB of variable *k* and the return value of the function. The value of data variation tends to be infinitely close to 0 as the algebraic *t* increases. Based on the above operations, the overall search of the operator in the data set is completed, and the IoT data information that meets the data mining requirements is output. Through all the above processing steps, the design of the IoT big data mining algorithm based on artificial intelligence technology is realized.

The article "Web Log Analysis and Security Assessment Method Based on Data Mining" was published in 2022. Journal: Comput Intell Neurosci.

### 3.3. Data Mining Based on Influencing Factors

In the data analysis based on influencing factors, this paper introduces the Gray Wolf Optimal Algorithm (GWO) in the field of data mining. The GWO algorithm is an optimization algorithm based on the gray wolf population hierarchy and group predation behavior. The principle is described in mathematical language as follows: For a gray wolf population, its number is *M*, and the search space is *k*, and for the gray wolf individual numbered *i*, its position can be described as

(12) $$\begin{array}{c} x_{i}=\left(x_{1},x_{2},\ldots x_{k}\right) \end{array}$$

(13) and (14) give the process of wolves surrounding their prey:

(13) $$\begin{array}{c} D=\left|C.x_{p}\left(t\right)-x\left(t\right)\right|, \end{array}$$

(14) $$\begin{array}{c} x\left(t+1\right)=x_{p}\left(t\right)-A\times D. \end{array}$$

Among them, *D* is the distance between the wolf and the prey in the wolf pack, *x*(*t*) is the individual position of the gray wolf after iteration, and *A* and *C* are the parameter vectors of the model. The calculation method is as follows:

(15) $$\begin{array}{c} A=2ar_{1}-a,\\ c=2r_{2}. \end{array}$$

When rank *α*, *β*, *δ* is close to the prey in the gray wolf group, the position of the prey can be estimated at this time, and the gray wolf group will iteratively update the position according to *α*, *β*, *δ*. Combined with the application scenarios in this paper, the common gray wolf optimization algorithm has a local optimum in the iterative process. Therefore, dynamic evolution operators and nonlinear convergence factors are introduced into the traditional gray wolf algorithm to improve the performance of the algorithm. After introducing the dynamic evolution operator, the wolf population combines the position of *α*, *β*, *δ* to update the position. At this point, the location update method can be rewritten as

(16) $$\begin{array}{c} \alpha =2-\left(e^{1/t}-1\right).\frac{2}{\left(e-1\right)}. \end{array}$$

Differential evolution algorithm is used in this paper when making evolution improvements to the improved gray wolf algorithm. The algorithm includes three steps of mutation, crossover, and selection. First, the population is initialized:

(17) $$\begin{array}{c} x_{ij}\left(0\right)=x^{L}{}_{ij}+r\text{and}\left(0,1\right)\left(x^{u}{}_{ij}-x^{L}{}_{ij}\right). \end{array}$$

Mutate *N* initial populations on a random search space:

(18) $$\begin{array}{c} V_{i}\left(t+1\right)=x_{r1}\left(t\right)+F\left[x_{r2}\left(t\right)-x_{r3}\left(t\right)\right]. \end{array}$$

Then perform a crossover operation to improve the diversity of the population:

(19) $$\begin{array}{c} U_{ij}\left(t+1\right)=X_{ij}\left(t+1\right). \end{array}$$

Based on the greedy algorithm, the individual with better evolution is selected as the new generation individual:

(20) $$\begin{array}{c} X_{ij}\left(t+1\right)=U_{i}\left(t+1\right),f\left[U_{i}\left(t\right)\right]\leq f\left[X_{i}\left(t\right)\right]. \end{array}$$

## 4. Web Log Analysis and Security Assessment under Data Mining

### 4.1. Web Log Security Assessment

In order to test the security performance of web logs, we collected the following data to evaluate the data coverage, accuracy, and recall to obtain the experimental results. The experimental results are shown in Table 1 and Figure 3.

According to the experimental data in the above chart, we can conclude that the accuracy rate and security score of web logs have reached more than 90%, and the coverage rate has reached 81%, and the recall rate is only 44%, while the accuracy rate and security score of ordinary logs have only reached about 80%, and the coverage rate is only 70%, and the recall rate reaches 57%. Through comparative experiments, we can see that web logs are more stable than ordinary logs in terms of coverage accuracy and security score.

The article "Web Log Analysis and Security Assessment Method Based on Data Mining" was published in 2022. Journal: Comput Intell Neurosci.

### 4.2. Overview of Web Log Hotspots and Trend Analysis

We have made comprehensive statistics on the hot issues mentioned in the web logs and counted the overall traffic, monthly hot spots, and the highest visiting days and traffic. The data obtained are shown in Table 2 and Figure 4.

As can be seen from the above figure, the number of visits was the highest in the fifth week, and the number of visits this week reached 99,473. The least week was the first week, with 87,655 visits. From the trend point of view, the fluctuation of the number of visits is dominated by a continuous upward trend, with a slight increase in the number of abnormal weekly visits.

#### 4.2.1. Web Log Hotspot Query Type

As shown in Figure 5 above, the largest query type was sales, which accounted for 33% of the total; by contrast, intermediaries had the lowest share, accounting for less than 20% of the total. This is followed by Ajax pages at 17% to 29%, followed by Ajax pages at 18% to 22%. In terms of trends, the sales page has maintained a high level of attention for a long time, while the data on the intermediate pages is scattered and incomplete, making it difficult to build a stable trend.

#### 4.2.2. Visits of Web Logs during Hot Spots

As can be seen from Figure 6 above, the hot spots browsed by users are all concentrated in the noon and June period, the frequency of visits reaches the highest and its proportion reaches about 15%, and the time period with the lowest visit frequency is 3. During the month, it accounted for about 7%. From the above figure, we can see that the time period of hotspot access is always fluctuating, and there is no stable trend.

### 4.3. Data Mining Accuracy Comparison

According to the experimental results, we can conclude that the data mining method used in this paper is relatively high in terms of experimental results and accuracy. The statistical method was compared, and the comparison results are shown in Figure 7.

According to the experimental data of the graph, we can know that the evaluation accuracy of the data mining method is the highest among the three methods. When the number of iterations reaches 50, the evaluation accuracy can reach 1, and when the number of iterations of the fuzzy statistical method is 80. When the number of iterations of the game method is 90, the evaluation accuracy can reach 1.

The article "Web Log Analysis and Security Assessment Method Based on Data Mining" was published in 2022. Journal: Comput Intell Neurosci.

### 4.4. Performance Test and Safety Evaluation Test

In order to test the superiority of the performance based on the data mining technology proposed in the paper, after the model proposed in the paper is improved, the fuzzy statistics method and the quantitative statistics method are, respectively, run on the test set and the mixed test set. The test set is used to evaluate the generalization ability of the final model, and the mixed test set is used to tune the model's hyperparameters and to make an initial evaluation of the model's ability. Record the experimental results to verify the advantages of the three methods, and draw graphs based on the experimental results. The experimental data of different models on the test set and the mixed test set are shown in Table 3 and 4.

According to the data in the table and Figure 8, we can conclude that, after running on the test set, the accuracy rate of quantitative statistics method can reach 89%, the accuracy rate can reach 91%, and the accuracy rate through data mining technology can reach 92.%, The accuracy rate can reach 93%, which is the highest index value among the three experimental models. The accuracy rate of fuzzy statistics method is 85%, which is the lowest among the three models. According to the curves of the three models, we can also see that the curve values of the data mining technology are very stable, the curve value of the quantitative statistics method is kept at about 0.90, and the curve value of the data mining method is also always kept at 0.97. The curve value of the statistical method is lower, and the experimental results also show that the performance of the data mining technology is the best and the security performance is also the best.

According to the data in Table 4 and Figure 9, we can conclude that, after running on the mixed test set, the performance of the three models has decreased to a certain extent, but the data mining method proposed in the article is still the highest among the three methods. One, the accuracy rate of quantitative statistics method is 87%, and the accuracy rate of fuzzy statistics method is 90%. According to the curves of the three algorithms, we can also see that the curve value of deep mining is very stable, whether in the test set or the mixed test set, the curve value has been kept at 0.95, and the curve of the fuzzy statistical method and the quantitative statistical method values stabilized within the range 0.90–095. The experimental results also show that the data mining method has the highest recognition accuracy and the best security performance.

## 5. Conclusion

One of the most important parts of the web indexing arena is the indexing of your blog. Web log extraction can use powerful data mining algorithms to systematically manage our logs on web servers and then learn accessibility or user preferences, in part based on settings and usage patterns. Website analytics and interactive website experience will be enhanced, and intelligent personalization will be provided to increase user loyalty. Through the analysis of the web log of data mining, we can also find that the curve value of deep mining is very stable no matter in the test set or the mixed test set, the curve value has been kept at 0.95, the curve value of fuzzy statistics method and quantitative statistics method is stable within the range of 0.90–095. The experimental results also show that the data mining method has the highest recognition accuracy and the best security performance.

The article "Web Log Analysis and Security Assessment Method Based on Data Mining" was published in 2022. Journal: Comput Intell Neurosci.

## Figures and Tables

**Figure 1:** Web log mining process.

**Figure 2:** Web data mining research objects.

**Figure 3:** Web log security assessment.

**Figure 4:** Week visits.

**Figure 5:** Hotspot query types.

**Figure 6:** Visits during hotspots.

**Figure 7:** Evaluation accuracy comparison test.

**Figure 8:** Curves on the test set.

**Figure 9:** Curves on the mixed test set.

**Table 1:** Web log security assessment.

Log model	Coverage (%)	Accuracy (%)	Recall (%)	Safetyscore (%)
Web log	81	93	44	94
Normal log	70	83	57	82

**Table 2:** Weekly visits.

	First	second	Third	Fourth	Fifth
Weekly visits	87655	87898	88242	89883	99473

**Table 3:** The performance of each model on the test set.

Method	Accuracy (%)	Accuracy (%)	Score (%)
Data mining	92	93	95
Fuzzy statistics	85	82	83
Quantitative statistics	89	91	90

**Table 4:** The performance of each method on the mixed test set.

Method	Accuracy (%)	Accuracy (%)	Score (%)
Quantitative statistics	87	88	90
Data mining	90	92	95
Fuzzy statistics	82	81	85

## Data Availability

The experimental data used to support the findings of this study are available from the corresponding author upon request.
